The article "MicroRNA‐140‐5p elevates cerebral protection of dexmedetomidine against hypoxic–ischaemic brain damage via the Wnt/β‐catenin signalling pathway" was retracted in 2021. Reasons: fabricated or falsified data; manipulated images; an official misconduct investigation; misconduct by an author.

# MicroRNA‐140‐5p elevates cerebral protection of dexmedetomidine against hypoxic–ischaemic brain damage via the Wnt/β‐catenin signalling pathway

**DOI:** 10.1111/jcmm.13597

**Published:** 2018-03-13

**Authors:** Xin‐Rui Han, Xin Wen, Yong‐Jian Wang, Shan Wang, Min Shen, Zi‐Feng Zhang, Shao‐Hua Fan, Qun Shan, Liang Wang, Meng‐Qiu Li, Bin Hu, Chun‐Hui Sun, Dong‐Mei Wu, Jun Lu, Yuan‐Lin Zheng

**Affiliations:** ^1^ Key Laboratory for Biotechnology on Medicinal Plants of Jiangsu Province School of Life Science Jiangsu Normal University Xuzhou Jiangsu Province China; ^2^ College of Health Sciences Jiangsu Normal University Xuzhou Jiangsu Province China

**Keywords:** cerebral protection, dexmedetomidine, hypoxic–ischaemic brain damage, micriRNA‐140‐5p, Wnt/β‐catenin signalling pathway, Wnt1

## Abstract

Hypoxia–ischaemia (HI) remains a major cause of foetal brain damage presented a scarcity of effective therapeutic approaches. Dexmedetomidine (DEX) and microRNA‐140‐5p (miR‐140‐5p) have been highlighted due to its potentially significant role in the treatment of cerebral ischaemia. This study was to investigate the role by which miR‐140‐5p provides cerebral protection using DEX to treat hypoxic–ischaemic brain damage (HIBD) in neonatal rats via the Wnt/β‐catenin signalling pathway. The HIBD rat models were established and allocated into various groups with different treatment plans, and eight SD rats into sham group. The learning and memory ability of the rats was assessed. Apoptosis and pathological changes in the hippocampus CA1 region and expressions of the related genes of the Wnt/β‐catenin signalling pathway as well as the genes responsible of apoptosis were detected. Compared with the sham group, the parameters of weight, length growth, weight ratio between hemispheres, the rate of reaching standard, as well as Bcl‐2 expressions, were all increased. Furthermore, observations of increased levels of cerebral infarction volume, total mortality rate, response times, total response duration, expressions of Wnt1, β‐catenin, TCF‐4, E‐cadherin, apoptosis rate of neurons, and Bax expression were elevated. Following DEX treatment, the symptoms exhibited by HIBD rats were ameliorated. miR‐140‐5p and si‐Wnt1 were noted to attenuate the progression of HIBD. Our study demonstrates that miR‐140‐5p promotes the cerebral protective effects of DEX against HIBD in neonatal rats by targeting the Wnt1 gene through via the negative regulation of the Wnt/β‐catenin signalling pathway.

## 1 INTRODUCTION

Hypoxic–ischaemic brain damage (HIBD) represents a commonly occurring life‐threatening disorder in the neonatal period, which is also observed in patients with stroke or cardiac arrest.^1^, ^2^ HIBD leads to permanent brain damage in infants and is frequently accompanied by various disabilities, such as cerebral palsy (10% infants), cognitive disorders (25%‐50% infants), learning disabilities and epilepsy.^3^, ^4^ HIBD, caused either in part or by total cerebral hypoxia, cerebral blood flow reduction and suspensions, is widely regarded as a key factor in central nervous system diseases.^5^ A progressive increase in the incidence and mortality rate of HIBD has seen the rate increasing from 1 to 8 incidences per 1000 live births.^1^, ^6^ At present, treatment options are confined to supportive care due to the complex mechanism and severity of the condition.^7^ In addition, previous studies have provided evidence suggesting that microRNAs (miRNAs) are aberrantly expressed in the tissues of rat models with ischaemic stroke, such as miR‐140.^8^ Thus, it is feasible to explore the highlighting the clinical research value of miRNAs and the unearthing the underlying mechanism behind HIBD in neonatal rats.

miRNAs refer to small non‐coding RNA molecules, which have been linked to tumour progression and carcinogenesis by targeting oncogenes or tumour suppressor genes.^9^ Previous studies have indicated decreased microRNA‐140‐5p (miR‐140‐5p) expression to be a common factor among human cancers combined with a reduction in cell migration and invasion, asserting that miR‐140‐5p could be a tumour suppressor gene.^10^ Furthermore, miR‐140 expression is notably decreased after HIBD. In addition, studies have revealed miR‐140‐5p plays an essential angiogenesis role in the ischaemia model via its regulation of VEGFA, which may be beneficial for cerebral ischaemia treatment.^8^ The combination of miRNAs reduction and Wnt/β‐catenin signalling pathway could promote cancer metastasis, carcinogenesis and even drug resistance.^11^ Reports have indicated that the mechanism of cell apoptosis is involved in the pathogenesis of nerve injury following the occurrence of hypoxia–ischaemia, suggesting that anti‐apoptotic actions could reverse neuronal damage.^12^, ^13^ The Wnt/β‐catenin signalling pathway plays a central role in hypoxia–ischaemia (HI) as well as in other neurodegenerative disorders, thus revealing a potential target for the treatment of HIBD.^14^ Dexmedetomidine (DEX) has been reported to up‐regulate the blood pressure and heart rate, as well as down‐regulating HIBD.^15^ Therefore, the central aim of our study was to explore the effect of miR‐140‐5p by targeting Wnt1 through the Wnt/β‐catenin signalling pathway in relation to the cerebral protection role of DEX from HIBD in neonatal rats.

The article "MicroRNA‐140‐5p elevates cerebral protection of dexmedetomidine against hypoxic–ischaemic brain damage via the Wnt/β‐catenin signalling pathway" was retracted in 2021. Reasons: fabricated or falsified data; manipulated images; an official misconduct investigation; misconduct by an author.

## 2 MATERIALS AND METHODS

### 2.1 Ethical statement

All experimental procedures were conducted in strict adherence with the international guidelines and principles for Laboratory Animal Care. All animal experiments were conducted under the ethical approval of the Institutional Review Board (IRB) of Key Laboratory for Biotechnology on Medicinal Plants of Jiangsu Province, School of Life Science, Jiangsu Normal University.

### 2.2 HIBD model establishment of neonatal rats

A total of 175 neonatal Sprague Dawley (SD) rats (1‐week‐old, weighing 12‐16 g) both male and female, obtained from the Laboratory Animal Center of Key Laboratory for Biotechnology on Medicinal Plants of Jiangsu Province, School of Life Science, Jiangsu Normal University, were housed in a controlled environmental setting with regulated temperatures (20‐25°C), humidity (40%‐70%) and indoor wind speed (0.1‐0.2 m/s). HI was conducted in the neonatal rats. The specific steps of HIBD model 16 establishment are described as follows: SD rats of 7 days were anaesthetized via ethyl ether inhalation and fixed in the supine position on a small operation table. Then, neck skin was cut open, and the left carotid artery was ligated, followed by incision suturing. After resting for 2 hour, the rats were placed in a hermetic organic glass box (5000 mL), with gas mixture containing 8% oxygen passing through (flow rate of 3 L/min). Normal oxygen supply was performed 2 h later. The rats which turned left or turned left with tail after HI were enrolled in the subsequent experiments.^17^ In total, 169 rats were successfully modelled.

### 2.3 Animal grouping and treatment

A total of eight neonatal SD rats, aged 1 week, free of HI were randomly selected as sham group that were provided by the Laboratory Animal Center of Key Laboratory for Biotechnology on Medicinal Plants of Jiangsu Province, School of Life Science, Jiangsu Normal University. The 169 HIBD rat models were assigned randomly into seven groups, namely the model group (eight rats), DEX group (23 rats, injected with DEX), miR‐140‐5p mimic (23 rats), DEX + negative control (NC) group (23 rats), DEX + miR‐140‐5p mimic group (23 rats), DEX + miR‐140‐5p inhibitor group (23 rats), DEX + si‐Wnt1 group (low expression of Wnt1, 23 rats) and DEX + miR‐140‐5p inhibitor + si‐Wnt1 group (23 rats). The treatment administered to each group was as follows: a small incision was made to the neck region of rats in the sham group without ligation, and the rats were provided with normal air for ventilation after suturing the incision, followed by an injection of 100 μL normal saline (0.1 mg/kg). The remaining groups were all treated according to the HIBD model establishment. In the DEX group, the HIBD model rats were injected intraperitoneally with 100 μL DEX (No. H20090248, 0.1 mg/kg, Jiang Su Heng Rui Pharmaceutical Co, Ltd., Lianyungang, Jiangsu, China) immediately after HI. In the miR‐140‐5p mimic group, rats were injected intravenously with 50 nmol/L miR‐140‐5p mimic immediately after HI. In the DEX + NC group, rats were injected intraperitoneally with 100 μL DEX (0.1 mg/kg), injected intravenously with the mixture (100 μL) of miR‐140‐5p mimic NC (No. miR01201‐1‐5, 50 nM, Ribobio Biological Technology Co. Ltd., Guangzhou, Guangdong, China) and Lipo 2000 (20 nmol/L) immediately after HI. In the DEX + miR‐140‐5p mimic group, rats were intraperitoneally injected with 100 μL DEX (0.1 mg/kg) and injected intravenously with the mixture (100 μL) of miR‐140‐5p mimic and Lipo 2000 (20 nmol/L) immediately after HI. In the DEX + miR‐140‐5p inhibitor group, rats were intraperitoneally injected with 100 μL DEX (0.1 mg/kg), injected intravenously with the mixture (100 μL) of miR‐140‐5p inhibitor (No. miR1000408‐1‐5, 50 nmol/L, Ribobio Biological Technology Co. Ltd., Guangzhou, Guangdong, China) and Lipo 2000 (20 nmol/L) immediately after HI. In the DEX + si‐Wnt1 group, the rats were injected intraperitoneally with 100 μL DEX (0.1 mg/kg), injected intravenously with the mixture of si‐Wnt1 (100 μmol/L) and Lipo 2000 (20 nmol/L) immediately after HI. In the DEX + miR‐140‐5p inhibitor + si‐Wnt1 group, rats were injected intraperitoneally with 100 μL DEX (0.1 mg/kg), injected intravenously with the mixture (100 μL) of miR‐140‐5p inhibitor (50 nmol/L), si‐Wnt1 (100 μmol/L) and Lipo 2000 (20 nmol/L) immediately after HI. In accordance with the aforementioned procedure, a series of injections were administered to each group, once a day for 3 days. Weight and growth rates were recorded.

The article "MicroRNA‐140‐5p elevates cerebral protection of dexmedetomidine against hypoxic–ischaemic brain damage via the Wnt/β‐catenin signalling pathway" was retracted in 2021. Reasons: fabricated or falsified data; manipulated images; an official misconduct investigation; misconduct by an author.

### 2.4 Y maze method

The respective learning and memory abilities of rats were detected using the Y maze method. After 3 days, five surviving rats were randomly selected from the sham and model groups, while 10 surviving rats were selected from other groups. While being assessed, the phenomenon that rats directly jumped to the safety zone after receiving electric shock was regarded to be the correct response, and the opposite was regarded as a wrong response. When nine correct responses occurred after 10 consecutive electric shocks, the rats were presumed to have achieved the “learnt” standard. The test was conducted again to reobserve memory ability after 24 hour. If rats did not reach the standard in the first or second test, no other statistical analyses were conducted except the rate of reaching standard. The specific standards were described as follows: (i) the rate of reaching standard: each training session was limited to 60 sequences and that learning well within 60 sequences indicating the rats had reached the standard; (ii) the response times before reaching the standard; (iii) the total response time was regarded as the sum of time in each response, which was calculated from the beginning of signal lamp to rats entering the safety zone; (iv) the response rate of active avoidance meant the percentage of response times in 5 second of the total response times; (5) the rate of correct response meant the percentage of correct response times and the total response times.

### 2.5 Determination of weight and water content of cerebral hemisphere

Three surviving rats were randomly selected from the sham and model groups, and ten surviving rats were selected from the other remaining groups (a total of 76 rats). Next, the rats were decapitated and their brains were obtained to observe the morphological changes of the left hemisphere with the naked eye. The left and right hemispheres of rats were then cut open through the midline. The wet weights of the hemispheres were recorded before baking in the oven at 80°C, and after 24 hour had elapsed, the dry weights were recorded. The degree of atrophy in the left hemisphere was determined by the wet weight ratio of left hemisphere to the right hemisphere, while the degree of oedema was determined by the water content rate. The water content rate was calculated according to the following formula (%) = (wet weight – dry weight)/wet weight × 100.

### 2.6 2,3,5‐triphenyltetrazolium chloride (TTC) staining

Sections of hippocampus tissues in each group were selected and placed into a newly prepared 2% TTC solution, followed by an incubation period in water bath without light exposure at 37°C for 30 minutes. After the colour had completely developed, the sections were fixed in 10% formaldehyde for a minimum of 24 hour and stored in the dark. The normal tissues were red in colour after TTC staining, and the infarcted tissues appeared white. The fixed brain slices were photographed, and the photographs were uploaded to the computer. The images were analysed using the automatic image analysis system (IBSA 2.7). The approximate volume of the cerebral infarction was = (cerebral infarction volume/brain tissue volume) × 100%.

### 2.7 Haematoxylin–eosin (HE) staining

Three surviving rats were randomly selected from the sham and model groups, while ten surviving rats were selected from the other groups, respectively. After etherization, thoracotomy was conducted, with 4°C normal saline and 4% paraformaldehyde perfused. The rats were then decapitated and their brains were obtained, cut through the midpoint of the frontal lobe and optic chiasma, followed by an incision into the optic chiasma. The samples were stored, fixed in 10% neutral formaldehyde solution overnight and embedded in paraffin. Next, the sections were sliced sequentially, and HE staining was conducted to observe cytomorphology under a light microscopy. The remaining slices were reserved for further use. The procedures for HE staining were conducted according to the following procedure. The sections were dewaxed twice in xylene (5‐15 min for each time) and dehydrated in anhydrous ethanol (100%, 95%, 80% and 75%, each for 1 min, respectively) twice. After rinsing using tap water for 3 min, the sections were stained with haematoxylin for 8 minute. After rinsing using tap water for 5 min, the sections were stained using eosin solution for a period of 2 minute, and then routinely dehydrated, cleaned and mounted in neutral balsam. The cytomorphological changes were observed under a microscope with high magnification.

The article "MicroRNA‐140‐5p elevates cerebral protection of dexmedetomidine against hypoxic–ischaemic brain damage via the Wnt/β‐catenin signalling pathway" was retracted in 2021. Reasons: fabricated or falsified data; manipulated images; an official misconduct investigation; misconduct by an author.

### 2.8 Nissl staining

The section samples in each group were collected. Nissl staining was conducted after the sections were dewaxed and rehydrated. The sections were stained using 0.1% toluidine blue at 60°C for 1 min and then washed under running water. Next, the sections were dehydrated and dissimilated in 95% ethanol under a microscope, followed by dehydration, permeabilizing and sealing. Numbers of neuron (per unit) in the hippocampal CA1 region were counted under a light microscope (×400).

### 2.9 Terminal deoxynucleotidyl transferase‐mediated dUTP‐biotin nick end labelling (TUNEL) assay

The sections of rat hippocampus tissues in each group were collected and TUNEL staining was conducted based on the instructions of the TUNEL kit (Roche, Basel, Switzerland). Paraffin‐embedded sections were baked at 60°C for 15 minute. The sections were dewaxed with xylene and then rehydrated using gradient ethanol. The sections were treated with proteinase K for 10 min and washed with PBS three times. TUNEL reacted solution was then prepared (TdT: mixture of nucleic acid = 1:9) and added to the sections for incubation at 37°C for 1 hour. The sections were treated with methanol containing 3% H_2_O_2_ at room temperature and washed with PBS three times. Converting peroxidase solution was then added to the sections and incubated at 37°C for 30 minute, followed by three PBS washes. The sections were developed by diaminobenzidine and washed again with PBS. Later the nuclei in sections were recoloured by haematoxylin and sections were dehydrated by gradient ethanol, followed by clearing with xylene and sealing with neutral gum. Cells with a brown nucleus were considered to be positive cells (which were observed under a light microscope), and the nuclei of the positive cells as well as the morphology of the cytoplasm were observed and recorded.

The article "MicroRNA‐140‐5p elevates cerebral protection of dexmedetomidine against hypoxic–ischaemic brain damage via the Wnt/β‐catenin signalling pathway" was retracted in 2021. Reasons: fabricated or falsified data; manipulated images; an official misconduct investigation; misconduct by an author.

### 2.10 Reverse‐transcription quantitative polymerase chain reaction (RT‐qPCR)

Total RNA was extracted from a set of sections of brain sample and 293FT cells using the single‐step TRIzol method. RNase‐free water was used to dissolve RNA, and ND‐1000 ultraviolet–visible spectrophotometer (No. 30254725, Mettler‐Toledo GmbH, Greifensee, Switzerland) was applied to measure optical destiny (OD) value, in an attempt to determine the quality of the total RNA and to adjust the RNA concentration. The extracted RNA was reversely transcribed, and the reaction conditions were as follows: incubation at 70°C for 10 minute, ice bath for 2 minute, incubation at 42°C for 60 minute, at 70°C for 10 minute. The reversely transcribed cDNA were temporarily stored in a refrigerator at −20°C. The RT‐qPCR prime sequences are displayed in Table 1 using TaqMan probes.^18^ The reaction system was performed according to the instructions of TaqMan RT‐PCR kit (No. A15299, Thermo Fisher Scientific Inc, Beijing, China), and reaction conditions included pre‐denaturation at 95°C for 30 seconds, denaturation at 95°C for 10 seconds; annealing at 60°C for 20 seconds, and extension at 70°C for 10 seconds, which run for 40 cycles. A RT‐qPCR instrument (No. 0104016, Coyote Bioscience Co., Ltd, Beijing, China) was used to determine the relative mRNA expressions. U6 small nuclear RNA (snRNA) was applied as an internal control for miR‐140‐5p. β‐actin was the internal control for Wnt1, E‐cadherin, T cell factor 4 (TCF‐4), β‐catenin, B‐cell lymphoma‐2 (Bcl‐2) and Bcl‐2‐associated X protein (Bax). The relative quantification method was applied, and triplicate wells were set to reach the minimum cycle threshold (Ct) value, as well as to calculate the relative amount of mRNA copy number. The 2^−ΔΔCt^ method was used to indicate the relative expression multiples of mRNA.

**Table 1:** Primer sequences for RT‐qPCR

Target gene	Primer sequence
miR‐140‐5p	Forward: 5′‐CAGTGGTTTTACCCTATGGTAG‐3′
	Reverse: 5′‐ACCATAGGGTAAAACCACTGTT‐3′
U6	Forward: 5′‐GCTTCGGCAGCACATATACTAAAAT‐3′
	Reverse: 5′‐CGCTTCACGAATTTGCGTGTCAT‐3′
Wnt1	Forward: 5′‐GGACTTGCTTCTCTTCTCATAGCC‐3′
	Reverse: 5′‐CCACACAGGCATAGAGTGTCTGC‐3′
β‐catenin	Forward: 5′‐AAAATGGCAGTGCGTTTAG‐3′
	Reverse: 5′‐TTTGAAGGCAGTCTGTCGTA‐3′
E‐cadherin	Forward: 5′‐CGG TGG TCAAAGAGCCC TTAC T‐3′
	Reverse: 5′‐TGAGGG TTGGTGCAACAACG TCGTTA‐3′
TCF‐4	Forward: 5′‐CAGGATCCAAAAGCTGGTG‐3′
	Reverse: 5′‐CCGGATCCTATAAGACGG TGACGAG‐3′
β‐actin	Forward: 5′‐GCACCACACCTTCTACAATGAG‐3′
	Reverse: 5′‐ACAGCCTGGATGGCTACGT‐3′
Bcl‐2	Forward: 5′‐CTGGTGGACAACATCGCTCTG‐3′
	Reverse: 5′‐GGTCTGCTGACCTCACTTGTG‐3′
Bax	Forward: 5′‐CTGAGCTGACCTTGGAGC‐3′
	Reverse: 5′‐GACTCCAGCCACAAAGATG‐3′
Caspase‐3	Forward: 5′‐ATGGACAACAACGAAACCTC‐3′
	Reverse: 5′‐TTAGTGATAAAAGTACAGTTCTT‐3′

miR‐140‐5p, microRNA‐140‐5p; TCF‐4, T cell factor 4; Bcl‐2, B‐cell lymphoma‐2; Bax, Bcl‐2‐associated X protein; RT‐qPCR, reverse‐transcription quantitative polymerase chain reaction.

The article "MicroRNA‐140‐5p elevates cerebral protection of dexmedetomidine against hypoxic–ischaemic brain damage via the Wnt/β‐catenin signalling pathway" was retracted in 2021. Reasons: fabricated or falsified data; manipulated images; an official misconduct investigation; misconduct by an author.

### 2.11 Western blot analysis

Hippocampus sections of rats in each group or of the proteins extracted from the 293FT cells were selected, followed by the addition of 1× sodium dodecyl sulphate (SDS) lysate. The protein extraction was heated at 100°C for 5 minute. Next, 20 μL samples were uploaded onto 12% polyacrylamide gel for electrophoresis. β‐catenin protein was extracted from cytoplasm and karyon according to instructions of Nuclear and Cytoplasmic Protein Extraction kit (No. P0028, Beyotime Biotechnology Co., Ltd, Shanghai, China). After transferred to membrane, Tris‐buffered saline with Tween 20 (TBST) containing 5% bovine serum albumin (BSA) was supplemented to block proteins for 1 hour on a decolourizing shaking table. Following the removal of the blocking solution, the membrane was placed into a plastic groove, prepared with 5% BSA, Bcl‐2 antibody (ab692, Abcam, Inc, Cambridge, UK), Bax antibody (ab32503, Abcam, Inc, Cambridge, UK), cleaved caspase‐3 antibody (ab232, Abcam, Inc, Cambridge, UK), Wnt1 protein antibody (ab105740, Abcam, Inc, Cambridge, UK), β‐catenin protein antibody (ab32572, Abcam, Inc, Cambridge, UK), E‐cadherin protein antibody (ab1416, Abcam, Inc, Cambridge, UK), TCF‐4 protein antibody (ab185736, Abcam, Inc, Cambridge, UK) and β‐actin (ab8226, Abcam, Inc, Cambridge, UK) were supplemented and placed in a refrigerator at 4°C overnight with oscillation, during which the transferring surface was upward. The next day, TBST was used 3 times for washing purposes (10 minute per wash). Diluted secondary antibodies (Abcam, Inc, Cambridge, UK) were added for an incubation period of 4‐6 hour at 4°C according to the same procedures. After the membranes were washed using TBST three times (15 minute per wash), chemiluminescence reagents: solution A and solution B (No. JFDW0002, Beijing Jorferin Bio‐Technology Co., Ltd, Beijing, China), were mixed at a ratio of 1:1. Following this, the membranes were completely immersed in the chromogenic reagent for 1 minute. After an extra chromogenic reagent was blotted using filter paper, the membranes were placed evenly into a cassette to avoid bubble formation. The sections were placed onto the membrane devoid of light. The membranes were pressed for 30 seconds — 40 minute and adjusted according to the lightness. X‐ray film was taken out to develop for 20 seconds and then precipitated for 20 seconds, followed by washing and photographing. β‐catenin protein concentration of endochylema and karyon was measured by bicinchoninic acid (BCA) protein assay kit (No. P0009, Beyotime Biotechnology Co., Ltd., Shanghai, China). Other protein bands of Western blot analysis were analysed by means of gel electrophoresis imaging system (No. MSD‐2000, Msdyq Tech Co. Ltd., Beijing, China) on relative optical density (OD), and β‐actin protein was used to correct the differences in protein loading and/or transfer between the groups.

The article "MicroRNA‐140‐5p elevates cerebral protection of dexmedetomidine against hypoxic–ischaemic brain damage via the Wnt/β‐catenin signalling pathway" was retracted in 2021. Reasons: fabricated or falsified data; manipulated images; an official misconduct investigation; misconduct by an author.

### 2.12 Immunofluorescence assay

A set of rat hippocampus sections was collected and frozen (20 pm). The sections were floated in 4% paraformaldehyde fixation and then washed three times with 0.01 mol/L PBS (10 minute for each time). The sections were treated with 0.3% H_2_O_2_ for 15 minute and washed three times with 0.01 mol/L PBS (10 minute for each time) again. The sections were then incubated in 0.3% Triton X‐100 solution for 30 minute, and then the primary antibody β‐catenin was added into sections (1: 1000, ab8226), followed by incubating at 37°C for 2 hour. The sections were then allowed to stand in 4°C for 16‐24 hour and washed three times with 0.01 mol/L PBS (10 minute for each time). The secondary fluorescent antibody labelled by horseradish peroxidase (HRP) (ab6721) was added into the sections and then incubated at 37°C for 2 hour while the remaining sections stood at room temperature for 2‐4 hour. The sections were then washed three times with 0.01 mol/L PBS (10 minute for each time). After being fixed with 50% glycerol, the sections were observed under a fluorescence microscope and photographed. All groups had their respective corresponding negative control group, and sections in negative control groups were not added to the primary antibody. The remaining steps were the same; however, there was no positive control for each group.

### 2.13 Construction of 3′ untranslated region (UTR) reporter gene plasmid vector

Wnt1 was determined as the potential target gene of miR‐140‐5p, based on the target gene prediction analysis using the TargetScan prediction algorithm (Whitehead Institute for Biomedical Research, Cambridge, MA, USA) in addition to other existing researches.^19^ Human target gene sequences deposited in the GenBank database (National Center for Biotechnology Information, Bethesda, Maryland, USA) were searched, and the 3′‐UTR sequence containing the potential target gene Wnt1 of miR‐140‐5p was designed according to the prediction results. Reporter gene plasmid vector (No. GUR100014‐P‐2, Ribobio Biological Technology Co. Ltd., Guangzhou, Guangdong, China) containing Wnt1‐3′UTR wild type and Wnt1‐3′UTR mutant was constructed via one‐step site‐directed mutagenesis. A BamH I cleavage site was added in front of the Wnt1‐3′UTR sequence transcription initiation codon ATG. Through another EcoR I cleavage site coexistent with pcDNA3.1/PS1 plasmid, the synthesized Wnt1 3′‐UTR sequence was cloned into the multiple cloning sites of wild‐type and mutant pcDNA3.1/PS1 plasmid at the BamH I and EcoR I cleavage sites, respectively. Thus, a vector for co‐expression of wild‐type and mutant of PS1 and Wnt1 3′‐UTR sequences was constructed. The vector construction for protein co‐expression was later verified through the determination of the restriction endonuclease dual‐enzyme digestion.

The article "MicroRNA‐140‐5p elevates cerebral protection of dexmedetomidine against hypoxic–ischaemic brain damage via the Wnt/β‐catenin signalling pathway" was retracted in 2021. Reasons: fabricated or falsified data; manipulated images; an official misconduct investigation; misconduct by an author.

### 2.14 Dual‐luciferase reporter gene assay

Cultured 293FT cells were seeded into a 96‐well culture plate (4 × 10^4^ cells per well). When the cells had grown to between 80% and 90% confluency, they were transfected using Lipo 2000 reagent (No. 40802ES02, Yeasen Biotechnology Co. Ltd., Shanghai, China). The template DNA (0.2 μL/well, 2 μg/μL) and Lipo 2000 (0.5 μL/well) were mixed with 25 μL culture medium, respectively. After being left standing for a period of 15 minute, the mixture was added to the plate. The, cells were then assigned into six groups: the Wntl‐3′UTR‐WT (blank control + WT), Wntl‐3′UTR‐MT (blank control + MT), miR‐140‐5p mimic + Wnt1‐WT, mimic control + Wnt1‐WT, miR‐140‐5p mimic + Wnt1‐MT, mimic control + Wnt1‐WT groups. According to the cell grouping, corresponding miR‐140‐5p, plasmid vector, lipo2000 and internal control plasmid pRL‐TK were mixed gently and incubated at room temperature for 20 minute. The aforementioned mixture was added to the culture wells containing both cells and the medium, followed by gentle mixing. After this, the culture plate was placed in an incubator for incubation at 37°C. After transfection for 6 hour, the culture medium in the wells were discarded and replaced by serum‐containing MEM for further culture. After the cells had been transfected for 48 hour, dual‐luciferase reporter gene assay kit (No. E1960; Promega Biotech Co., Ltd, Madison, WI, USA) was conducted to measure the luciferase activity. After the cells had been transfected for 48 hour, the former medium was removed, and cells were washed twice using phosphate‐buffered saline (PBS). The cells in each well were then added with 100 μL passive lysis buffer (PLB) and shaken gently for 15 minute at room temperature. The cell lysates were subsequently collected. Using the program, 2 seconds was set for pre‐reading and 10 seconds was set for reading values, in which the volume of sample for uploading LARII and Stop&Glo Reagent was 100 μL. Next the prepared LARII and Stop&Glo Reagent were added into the luminescent tube or plate (20 μL of each sample) for detection by a bioluminescence fluorescence detector (No. 5210290, Labsystems, Helsinki, Finland).

The article "MicroRNA‐140‐5p elevates cerebral protection of dexmedetomidine against hypoxic–ischaemic brain damage via the Wnt/β‐catenin signalling pathway" was retracted in 2021. Reasons: fabricated or falsified data; manipulated images; an official misconduct investigation; misconduct by an author.

### 2.15 Statistical analysis

The SPSS 21.0 statistical software (SPSS Inc., Chicago, IL, USA) was applied to analyse the statistical data of the study. All the data were tested for normality. Measurement data were presented as mean ± standard deviation and tested for homogeneity of variances. The comparisons among multiple groups were conducted by the one‐way analysis of variance (ANOVA), while the comparisons between two groups with variance homogeneity were analysed by means of the least significant difference (LSD) or SNK (*q* test) test, and the comparisons between two groups without variance homogeneity were analysed by Tamhane's T2 test. A value of *P* < .05 indicated that the difference was of statistical significance.

## 3 RESULTS

### 3.1 The combined action of DEX and miR‐140‐5p blocks the Wnt/β‐catenin signalling pathway better than treated with DEX or miR‐140‐5p mimic alone

mRNA and protein expressions of Wnt/β‐catenin signalling pathway‐related genes of rats in each group are shown in Figure 1. Compared with the sham group, the expressions of miR‐140‐5p expression among rats were notably decreased in the model, DEX, miR‐140‐5p mimic, DEX + NC, DEX + miR‐140‐5p inhibitor, DEX + si‐Wnt1 and DEX + miR‐140‐5p inhibitor + si‐Wnt1 groups (all *P* < .05); however in the DEX + miR‐140‐5p mimic, no obvious difference from the sham group was observed (*P* > .05). The miR‐140‐5p expression of rats in the DEX, miR‐140‐5p mimic, DEX + NC, DEX + miR‐140‐5p mimic and DEX + si‐Wnt1 groups was higher than that in the model group (all *P* < .05). In comparison with the DEX group, the miR‐140‐5p expression of rats was reduced in the DEX + miR‐140‐5p inhibitor group; however, increased levels in the DEX + miR‐140‐5p mimic group were recorded (all *P* < .05). The mRNA and protein expressions of Wnt1, β‐catenin, TCF‐4 and E‐cadherin of rats in the model, DEX, miR‐140‐5p mimic, DEX + NC, DEX + miR‐140‐5p inhibitor and DEX + miR‐140‐5p inhibitor + si‐Wnt1 groups were all higher than those in the sham group (all *P* < .05), but not significantly different in the DEX + si‐Wnt1, DEX + miR‐140‐5p mimic groups from the sham group (all *P* > .05). Compared with the model group, mRNA and protein expressions of Wnt1, β‐catenin, TCF‐4 and E‐cadherin of the rats were decreased in the DEX, miR‐140‐5p mimic, DEX + NC, DEX + miR‐140‐5p mimic, DEX + si‐Wnt1 and DEX + miR‐140‐5p inhibitor + si‐Wnt1 groups (all *P* < .05). In comparison with the DEX group, mRNA and protein expressions of Wnt1, β‐catenin, TCF‐4 and E‐cadherin of rats were reduced in the DEX + miR‐140‐5p mimic and DEX + si‐Wnt1 groups, but those were increased in the DEX + miR‐140‐5p inhibitor group (all *P* < .05). Overexpressed miR‐140‐5p was demonstrated to be capable of suppressing the Wnt/β‐catenin signalling pathway in HIBD rats.

The article "MicroRNA‐140‐5p elevates cerebral protection of dexmedetomidine against hypoxic–ischaemic brain damage via the Wnt/β‐catenin signalling pathway" was retracted in 2021. Reasons: fabricated or falsified data; manipulated images; an official misconduct investigation; misconduct by an author.

**Figure 1:** The combined action of DEX and miR‐140‐5p suppresses the Wnt/β‐catenin signalling pathway detected by RT‐qPCR and Western blot analysis. Notes: A, Cartogram of miR‐140‐5p expression and mRNA expressions of Wnt/β‐catenin signalling pathway‐related genes (Wnt1, β‐catenin, TCF‐4 and E‐cadherin) of rats among eight groups; B, Cartogram of protein expressions of Wnt/β‐catenin signalling pathway‐related genes (Wnt1, β‐catenin, TCF‐4 and E‐cadherin) of rats among eight groups; C, Protein bands of Wnt/β‐catenin signalling pathway‐related proteins (Wnt1, β‐catenin, TCF‐4 and E‐cadherin) of rats among eight groups; D, Immunofluorescence staining image among eight groups *, *P* < .05, compared with the sham group; #, *P* < .05, compared with the model group; &, *P* < .05, compared with the DEX group; three surviving rats were randomly selected from each group; the experiment was repeated 3 times; DEX, dexmedetomidine; NC, negative control; miR‐140‐5p, microRNA‐140‐5p; TCF‐4, T cell factor 4

### 3.2 The combined action of miR‐140‐5p and DEX promotes weight and length growth of rats after treatment better than treated with DEX or miR‐140‐5p mimic alone

The parameters after treatment such as the growth conditions of weight and the length of rats in different groups are illustrated in Table 2. Compared with the sham group, the weight and length growth of rats was markedly decreased in the model, DEX, DEX + NC, DEX + miR‐140‐5p inhibitor and DEX + miR‐140‐5p inhibitor + si‐Wnt1 groups (all *P* < .05). In the DEX, miR‐140‐5p mimic, DEX + NC, DEX + miR‐140‐5p mimic, DEX + si‐Wnt1 and DEX + miR‐140‐5p inhibitor + si‐Wnt1 groups, the weight and length growth of rats was significantly increased when compared to the model group (all *P* < .05). Compared with the DEX group, the weight and length growth of rats was elevated in the DEX + si‐Wnt1 and DEX + miR‐140‐5p mimic groups; however, reductions were observed in the DEX + miR‐140‐5p inhibitor group (all *P* < .05). In comparison with the sham group, the indicators of rats, there were significant differences in the DEX + si‐Wnt1 and DEX + miR‐140‐5p mimic groups (*P* > .05). There was no obvious difference in relation to the indicators of rats between the model and DEX + miR‐140‐5p inhibitor groups (*P* > .05). The indicators of rats did not differ significantly among the DEX, DEX + NC, DEX + miR‐140‐5p inhibitor + si‐Wnt1 groups (*P* > .05).

The article "MicroRNA‐140‐5p elevates cerebral protection of dexmedetomidine against hypoxic–ischaemic brain damage via the Wnt/β‐catenin signalling pathway" was retracted in 2021. Reasons: fabricated or falsified data; manipulated images; an official misconduct investigation; misconduct by an author.

**Table 2:** Weight and length growth of rats after treatment among eight groups

Group	n	Weight growth (g)	Length growth (cm)
Sham group	8	6.23 ± 1.03	0.31 ± 0.03
Model group	23	3.12 ± 1.01*	0.13 ± 0.01*
DEX group	23	4.67 ± 1.11*, #	0.20 ± 0.03*, #
miR‐140‐5p mimic group	23	4.45 ± 1.11*, #	0.20 ± 0.03*, #
DEX + NC group	23	4.61 ± 1.12*, #	0.22 ± 0.04*, #
DEX + miR‐140‐5p mimic group	23	5.88 ± 1.11#, &	0.30 ± 0.03#, &
DEX + miR‐140‐5p inhibitor group	23	3.22 ± 1.08*, &	0.12 ± 0.01*, &
DEX + si‐Wnt1 group	23	5.84 ± 1.04#, &	0.29 ± 0.02#, &
DEX + miR‐140‐5p inhibitor + si‐Wnt1 group	23	4.68 ± 1.04*, #	0.20 ± 0.01*, #

The experiment was repeated three times.

DEX, dexmedetomidine; NC, negative control; miR‐140‐5p, microRNA‐140‐5p.

*P < .05, compared with the sham group; ^#^ *P* < .05, compared with the model group; ^&^ *P* < .05, compared with the DEX group.

### 3.3 The combined action of miR‐140‐5p and DEX promotes learning and memory ability of rats after treatment better than treated with DEX or miR‐140‐5p mimic alone

The result of the Y maze method demonstrated that the rate of reaching standard of rats in the sham group was 100%, and there was no significant difference in terms of the rate of reaching standard between the DEX + si‐Wnt1, DEX + miR‐140‐5p mimic and sham groups (*P* > .05), while the rate of reaching standard was found to be lower in all the other groups when compared with the sham group (*P* < .05). After two tests, no significant difference in total response times and duration, active avoidance and correct response rates was identified among the DEX + si‐Wnt1 and DEX + miR‐140‐5p mimic and sham groups (all *P* > .05). Rats in the sham group recorded significantly less total response times and duration than those in the model, DEX, miR‐140‐5p mimic, DEX + NC, DEX + miR‐140‐5p inhibitor and DEX + miR‐140‐5p inhibitor + si‐Wnt1 groups, while the active avoidance rate and correct response rate were higher than those in the other five groups (all *P* < .05). Compared with the model group, the total response times and duration of rats decreased after treated with DEX or miR‐140‐5p mimic, with the active avoidance and correct response rates all displaying increased levels (all *P* < .05), while miR‐140‐5p was shown to negatively influence the efficacy of si‐Wnt1 among HIBD rats (all *P* < .05) (Table 3).

**Table 3:** Learning and memory ability of rats after treatment among eight groups

Group		The first test				The second test			
	Rate of reaching standard (%)	Total response times	Total duration (s)	Active avoidance rate (%)	Correct response rate (%)	Total response times	Total duration (s)	Active avoidance rate (%)	Correct response rate (%)
Sham group (n = 5)	100 ± 0	16.91 ± 2.03	63.09 ± 5.81	68.32 ± 3.29	86.01 ± 6.01	10.02 ± 3.04	52.01 ± 4.24	78.49 ± 4.35	91.20 ± 4.93
Mode group (n = 10)	40.35 ± 4.32*	28.03 ± 3.09*	93.09 ± 7.03*	44.26 ± 2.01*	63.26 ± 5.82*	22.04 ± 2.38*	73.28 ± 5.02*	55.92 ± 245*	69.29 ± 4.98*
DEX group (n = 10)	76.42 ± 3.24*, #	23.42 ± 2.17*, #	77.13 ± 6.73*, #	55.24 ± 4.89*, #	74.82 ± 4.56*, #	15.98 ± 3.21*, #	65.25 ± 4.02*, #	66.32 ± 5.36*, #	78.93 ± 5.38*, #
miR‐140‐5p mimic group (n = 10)	75.39 ± 2.89	21.89 ± 1.89*, #	79.03 ± 5.03*, #	54.42 ± 4.72*, #	72.31 ± 4.27*, #	16.03 ± 2.01*, #	65.25 ± 4.32*, #	66.41 ± 3.2*, #	78.94 ± 4.32*, #
DEX + NC group (n = 10)	77.53 ± 3.68*, #	22.08 ± 2.18*, #	78.08 ± 5.93*, #	56.01 ± 4.27*, #	73.28 ± 3.71*, #	15.32 ± 2.89*, #	66.35 ± 4.92*, #	64.01 ± 3.89*, #	78.01 ± 5.03*, #
DEX + miR‐140‐5p mimic group (n = 10)	95.01 ± 2.41#, &	16.05 ± 2.09#, &	6.256 ± 5.33#, &	69.35 ± 4.82#, &	83.27 ± 5.24#, &	11.57 ± 2.71#, &	55.01 ± 3.2#, &	78.36 ± 4.82#, &	89.01 ± 5.39#, &
DEX + miR‐140‐5p inhibitor group (n = 10)	42.25 ± 1.52*, &	27.48 ± 2.87*, &	91.32 ± 7.15*, &	43.41 ± 3.72*, &	64.29 ± 4.62*, &	21.63 ± 2.01*, &	73.29 ± 3.51*, &	55.02 ± 3.29*, &	70.32 ± 4.39*, &
DEX + si‐Wnt1 group (n = 10)	96.32 ± 1.32#, &	16.82 ± 2.04#, &	67.25 ± 5.21#, &	65.92 ± 4.78#, &	82.46 ± .92#, &	10.43 ± 2.19#, &	57.02 ± 4.02#, &	76.34 ± 3.25#, &	88.32 ± 6.34#, &
DEX + miR‐140‐5p inhibitor + si‐Wnt1 group (n = 10)	74.21 ± 3.25*, #	23.36 ± 2 .17*, #	76.25 ± 5.27*, #	54.82 ± 4.25*, #	74.02 ± 3.82*, #	17.02 ± 3.82*, #	65.89 ± 2.14*, #	65.32 ± 4.31*, #	78.32 ± 5.12*, #

DEX, dexmedetomidine; NC, negative control; miR‐140‐5p, microRNA‐140‐5p. The experiment was repeated three times.

The article "MicroRNA‐140‐5p elevates cerebral protection of dexmedetomidine against hypoxic–ischaemic brain damage via the Wnt/β‐catenin signalling pathway" was retracted in 2021. Reasons: fabricated or falsified data; manipulated images; an official misconduct investigation; misconduct by an author.

*P < .05, compared the sham group; ^#^ *P* < .05, compared the model group; ^&^ *P* < .05, compared the DEX group.

### 3.4 The combined action of miR‐140‐5p and DEX promotes weight but reduces the water content of brain hemisphere in rats better than treated with DEX or miR‐140‐5p mimic alone

Compared with the sham group, the weight ratio between the left hemisphere and right hemisphere was lower, with the water content of the left hemisphere detected to be higher in the model, DEX, miR‐140‐5p mimic, DEX + NC, DEX + miR‐140‐5p inhibitor and DEX + miR‐140‐5p inhibitor + si‐Wnt1 groups (all *P* < .05). There was no significant difference regarding the weight ratio between the left hemisphere and the right hemisphere as well as regarding the water content in the left hemisphere among the sham group and the DEX + si‐Wnt1 or DEX + miR‐140‐5p mimic groups (all *P* < .05). The DEX, miR‐140‐5p mimic, DEX + NC, DEX + miR‐140‐5p mimic, DEX + si‐Wnt1 and DEX + miR‐140‐5p inhibitor + si‐Wnt1 groups all displayed a greater weight ratio of the left hemisphere in comparison to the right hemisphere, but lower water content of the left hemisphere than the model group (all *P* < .05). In comparison with the DEX group, the weight ratio between the left hemisphere and right hemisphere was increased, with the water content of left hemisphere exhibiting decreases in the DEX + miR‐140‐5p mimic and DEX + si‐Wnt1 groups; however, a contrasting trend was observed in the DEX + miR‐140‐5p inhibitor group (all *P* < .05) (Table 4).

**Table 4:** Brain weight and water content of rats among eight groups

Groups	n	Weight ratio of left hemisphere to right one	Water content of left hemisphere (%)
Sham group	3	1.03 ± 0.04	80.2 ± 0.5
Model group	3	0.69 ± 0.07*	89.9 ± 0.8*
DEX group	10	0.85 ± 0.08*, #	84.6 ± 0.7*, #
miR‐140‐5p mimic group	10	0.82 ± 0.08*, #	81.5 ± 0.7*, #
DEX + NC group	10	0.86 ± 0.08*, #	84.7 ± 0.5*, #
DEX + miR‐140‐5p mimic group	10	1.01 ± 0.05#, &	80.6 ± 0.4#, &
DEX + miR‐140‐5p inhibitor group	10	0.72 ± 0.06*, &	89.6 ± 0.6*, &
DEX + si‐Wnt1 group	10	0.99 ± 0.04#, &	80.9 ± 0.8#, &
DEX + miR‐140‐5p inhibitor + si‐Wnt1 group	10	0.85 ± 0.05*, #	84.3 ± 0.7*, #

DEX, dexmedetomidine; NC, negative control; miR‐140‐5p, microRNA‐140‐5p. The experiment was repeated three times.

*P < .05, compared with the sham group; ^#^ *P* < .05, compared with the model group; ^&^ *P* < .05, compared with the DEX group.

### 3.5 The combined action of miR‐140‐5p and DEX as well as si‐Wnt1 decreases cerebral infarction volume better than treated with DEX or miR‐140‐5p mimic alone

After TTC staining, the normal brain tissues were red in colour, with the infarction location displayed in white. There was no infarction in rats among the sham group, as well as varying degrees of infarctions in penumbra in the injured side of rats in the HIBD groups. Compared with the model group, infarctions in the DEX, miR‐140‐5p mimic, DEX + NC, DEX + miR‐140‐5p inhibitor + si‐Wnt1, DEX + si‐Wnt1 and DEX + miR‐140‐5p mimic groups decreased. Compared with the model group, in the DEX + si‐Wnt1 and DEX + si‐Wnt1 groups, cerebral infarction volume significantly decreased (*P* < .01). In the DEX, miR‐140‐5p mimic, DEX + NC and DEX + miR‐140‐5p inhibitor + si‐Wnt1 groups, cerebral infarction volume was smaller than that in the model group, but still larger than that in the DEX + si‐Wnt1, DEX + miR‐140‐5p mimic groups (all *P* < .05). There was no statistical significance detected in relation to the cerebral infarction volume between the DEX + miR‐140‐5p inhibitor and model groups (Figure 2A‐C). Overexpressed miR‐140‐5p and underexpressed Wnt1 were demonstrated to reduce cerebral infarction volume.

The article "MicroRNA‐140‐5p elevates cerebral protection of dexmedetomidine against hypoxic–ischaemic brain damage via the Wnt/β‐catenin signalling pathway" was retracted in 2021. Reasons: fabricated or falsified data; manipulated images; an official misconduct investigation; misconduct by an author.

**Figure 2:** The combined action of miR‐140‐5p and DEX as well as silencing of Wnt1 reduces cerebral infarction volume by TTC staining. Note: A, TTC staining of brain tissue of rats; B, cerebral infarction volume of rat brain tissues; C, area of cerebral infarction of rat brain tissues; *, *P* < .05, compared with the sham group; #, *P* < .05, compared with the model group; &, *P* < .05, compared with the DEX group; three surviving rats were randomly selected from the sham and model groups, respectively, and ten surviving rats were selected from other groups, respectively; the experiment was repeated three times; miR‐140‐5p, microRNA‐140‐5p; DEX, dexmedetomidine; NC, negative control; TTC, 2,3,5‐triphenyltetrazolium chloride

### 3.6 The combined action of miR‐140‐5p and DEX plays a promoting role in forming pyramid neurons of hippocampal CA1 region in the left hemisphere better than treated with DEX or miR‐140‐5p mimic alone

HE staining results revealed that neurons in the CA1 region exhibited clear layers, normal morphology and size, clear karyon, visible nucleolus, clear boundary of cell cluster, cytoplasm stained with light red, as well as densely arranged pyramid neurons. Compared with the sham group, neurons in the model group were observed to be slightly irregular in terms of their arrangement and morphology, swelling cells, part of hypochromatic karyon and cytoplasm weakly stained, even vesicular cells and karyopyknosis of some cells. In the DEX, miR‐140‐5p mimic, DEX + NC and DEX + miR‐140‐5p inhibitor + si‐Wnt1 groups, the neurons displayed essentially regular arrangements, with some swelling among the cells and karyopyknosis of some karyons and cell bodies. The DEX + si‐Wnt1 and DEX + miR‐140‐5p mimics groups and the sham group had similar cell arrangement in hippocampal CA1 region. In the DEX + miR‐140‐5p inhibitor group, neurons in the CA1 region had disorderly arrangement, some broken pyramid neurons, anachromasis karyon with strong staining and less normal neurons and pyramidal neurons had similar changes. See Figure 3A for details.

**Figure 3:** The combined action of miR‐140‐5p and DEX protects neurons of hippocampal CA1 region in the left hemisphere observed by HE staining and Nissl staining. Notes: A, HE staining of pyramid neurons in the hippocampal CA1 region of the left hemisphere (200×) & (400×); B, Nissl staining in the hippocampal CA1 region (400×); three surviving rats were randomly selected from the sham and model groups, respectively, and ten surviving rats were selected from other groups, respectively; the experiment was repeated three times; DEX, dexmedetomidine; NC, negative control; miR‐140‐5p, microRNA‐140‐5p; HE, haematoxylin eosin

The Nissl staining results revealed in the sham group, the structure of hippocampal CA1 region was clear, and cell morphology was normal in and more uniform in order, as well as the plaque like Nissl body appearing dark blue with a large amount of distribution. In the model group, the structure of hippocampal CA1 region was vague, cell number was decreased and cell was swelling was discrete in order, in addition to what appeared to be the dissolving of the Nissl body as well as vacuolization, and numbers of Nissl bodies were disappeared. Compared with the model group, in the DEX, miR‐140‐5p mimic, DEX + NC, DEX + miR‐140‐5p inhibitor + si‐Wnt1, DEX + si‐Wnt1 and DEX + miR‐140‐5p mimic groups, swelling and vacuolization of the cells were not of a significant degree of the number of missing Nissl body decreased. In the DEX + si‐Wnt1, DEX + miR‐140‐5p mimic groups, the number of missing Nissl bodies had significantly decreased. In the DEX, DEX + NC group and DEX + miR‐140‐5p inhibitor + si‐Wnt1 groups, the number of missing Nissl bodies was partially decreased; however, the number was still superior in comparison with the DEX + si‐Wnt1, DEX + miR‐140‐5p mimic groups. There was no significant difference in relation to the degree of swelling and vacuolization of cells as well as the number of missing Nissl bodies between the DEX + miR‐140‐5p inhibitor and model groups (Figure 3B).

The article "MicroRNA‐140‐5p elevates cerebral protection of dexmedetomidine against hypoxic–ischaemic brain damage via the Wnt/β‐catenin signalling pathway" was retracted in 2021. Reasons: fabricated or falsified data; manipulated images; an official misconduct investigation; misconduct by an author.

Staining results of the DEX + miR‐140‐5p mimic, DEX, miR‐140‐5p mimic and DEX + miR‐140‐5p inhibitor groups were indicative of the notion that miR‐140‐5p could slow the development of HIBD, while the inhibitors of miR‐140‐5p could reverse the protection like effects of si‐Wnt1 against HIBD. Staining results of the DEX and DEX + si‐Wnt1 groups indicated that the Wnt1 pathway cascade could promote the progression of HIBD. Overall, overexpressed miR‐140‐5p with DEX was revealed to protect neurons against HIBD.

### 3.7 The combined action of miR‐140‐5p and DEX inhibits cell apoptosis in HIBD rats better than treated with DEX or miR‐140‐5p mimic alone

TUNEL staining results (Figure 4A) indicated that, when compared with the sham group, cell apoptosis rate was elevated in the model, DEX, DEX + NC, DEX + miR‐140‐5p inhibitor and DEX + miR‐140‐5p inhibitor + si‐Wnt1 groups (all *P* < .05). There was no significant difference between the DEX + si‐Wnt1 and DEX + miR‐140‐5p mimic groups (*P* > .05). After HIBD rats were treated with DEX, miR‐140‐5p mimic and si‐Wnt1, the cell apoptosis rate was decreased; however, the miR‐140‐5p inhibitor was shown to reverse the protection of si‐Wnt1 against HIBD rats.

The article "MicroRNA‐140‐5p elevates cerebral protection of dexmedetomidine against hypoxic–ischaemic brain damage via the Wnt/β‐catenin signalling pathway" was retracted in 2021. Reasons: fabricated or falsified data; manipulated images; an official misconduct investigation; misconduct by an author.

**Figure 4:** The combined action of miR‐140‐5p and DEX dampens neuron apoptosis in HIBD rats. Notes: A, Results of TUNEL staining among groups; B, Histogram of cell apoptosis rate; C, mRNA expressions of apoptosis‐related genes; D, Protein expressions of apoptosis‐related genes; E, Protein bands of apoptosis‐related genes; *, *P* < .05, compared with the sham group; #, *P* < .05, compared with the model group; &, *P* < .05, compared with the DEX group; three surviving rats were randomly selected from the sham and model groups, respectively, and ten surviving rats were selected from other groups, respectively; the experiment was repeated three times; DEX, dexmedetomidine; NC, negative control; miR‐140‐5p, microRNA‐140‐5p; Bcl‐2, B‐cell lymphoma‐2; Bax, Bcl‐2‐associated X protein; TUNEL, terminal deoxynucleotidyl transferase‐mediated dUTP‐biotin nick end labelling

Compared with the sham group, there were no significant differences detected in regard to the expression of Bcl‐2 and Bax, caspase‐3 mRNA levels and cleaved caspase‐3 expression between the DEX + si‐Wnt1 and DEX + miR‐140‐5p mimic groups, with decreases in the expression of Bcl‐2, as well as the expression of Bax, caspase‐3 mRNA levels and cleaved caspase‐3 expression increased in other groups. After being treated with DEX and si‐Wnt1, the expression of Bcl‐2 increased, while expressions of Bax and mRNA level of caspase‐3 decreased in HIBD rats, with miR‐140‐5p inhibitor exhibiting its capability in the reversal of the protection of si‐Wnt1 against HIBD rats (Figure 4B‐E). Overexpressed miR‐140‐5p with DEX was found to protect neurons against apoptosis in HIBD rats.

### 3.8 Wnt1 is determined as the target gene of miR‐140‐5p

Wnt1 gene and corresponding target sites binding with miR‐140‐5p were predicted using the online prediction software of Target Scan (Figure 5A). The detection results of the dual‐luciferase reporter gene revealed that the luciferase activity of reporter gene was markedly decreased in the miR‐140‐5p mimic + Wnt1‐WT group (*P* < .05), while observations of the mutant groups revealed there to be no significant differences (all *P* > .05), when compared with the mimics control + Wnt1‐WT and blank control + Wnt1‐WT groups (Figure 5B). miR‐140‐5p negatively mediated Wnt1.

**Figure 5:** Wnt1 is verified as one of the target gene of miR‐140‐5p determined by dual‐luciferase reporter gene assay. Notes: A, Sequences in the 3′UTR of Wnt1 mRNA binding with miR‐140‐5p; B, Relative luciferase activity of Wnt l‐3′UTR reporter gene vector; *, *P* < .05, compared the mutant groups; the experiment was repeated three times; WT, wild type; MT, mutant; miR‐140‐5p, microRNA‐140‐5p

The article "MicroRNA‐140‐5p elevates cerebral protection of dexmedetomidine against hypoxic–ischaemic brain damage via the Wnt/β‐catenin signalling pathway" was retracted in 2021. Reasons: fabricated or falsified data; manipulated images; an official misconduct investigation; misconduct by an author.

### 3.9 miR‐140‐5p inhibits the expression of Wnt1 in 293FT cells

The result of RT‐qPCR and Western blot analysis suggested that the overexpression of miR‐140‐5p decreased the mRNA and protein expression of Wnt1, while the underexpression of miR‐140‐5p increased the mRNA and protein expression of Wnt1 in 293FT cells (*P* < .05) (Figure 6). miR‐140‐5p negatively regulated the expression of Wnt1. Overexpressed miR‐140‐5p demonstrated an ability to depress the expressions of Wnt1.

**Figure 6:** Overexpressed miR‐140‐5p inhibits the expression of Wnt1 in 293FT cells by RT‐qPCR and Western blot analysis. Notes: A, the histogram of mRNA expression of Wnt1; B, the histogram of the protein expression of Wnt1 and corresponding protein bands. *, *P* < .05, compared the control groups; the experiment was repeated three times

## 4 DISCUSSION

As a severe life‐threatening disease, HIBD largely contributes to incidences of permanent brain damage among infants, frequently resulting in disabilities of a high modality.^1^, ^3^ The abnormal expression of miR‐140 has been reported to be induced after HIBD. DEX has been proven to regulate HIBD.^8^, ^15^ In an attempt to elucidate a potential HIBD therapeutic target, an investigation was pursued into miR‐140‐5p and its effects on cerebral protection of DEX against HIBD by targeting Wnt1 through the Wnt/β‐catenin signalling pathway in neonatal rats.

During this study, a key finding revealed that miR‐140‐5p targeted and inhibited the Wnt1 gene, highlighting the negative regulation of the Wnt/β‐catenin signalling pathway. When compared with the model group, the expressions of miR‐140‐5p were increased in the DEX, DEX + NC, DEX + miR‐140‐5p mimic and DEX + si‐Wnt1 groups. A rat model of HIBD was successfully established according to the prescribed method in our procedure, which demonstrated that the neuroprotective effect in treating HIBD could be achieved via placenta‐derived mesenchymal stem cells through relieving oxidative stress.^3^ Several miR‐140‐5p targets are connected through the Wnt signalling pathway such as GPR177 and FZD6, which could reduce Wnt3a and Wnts expressions, largely suggesting that miR‐140‐5p could inhibit Wnt1 expression.^20^ Wnt signalling can be suppressed through antagonistic molecules such as Wnt inhibitory factor 1, while miRNAs have been reported to suppress the Wnt pathway by modulating β‐catenin.^11^ GPR177 has been demonstrated as being a Wnt transcriptional target essential for the secretion of Wnt, allowing miR‐140‐5p to also target Wnt1.^21^, ^22^, ^23^ Previous reports have indicated that Fzd6, which is generally regarded to be a receptor in the Wnt pathway as belonging to a negative regulator of the Wnt/β‐catenin signalling pathway, suggesting miR‐140‐5p could target the Wnt gene and regulate the Wnt/β‐catenin signalling pathway negatively.^24^ Similarly, miR‐142‐3p has been reported to down‐regulate Wnt/β‐catenin signalling, which is largely in line with the central findings presented in this study.^25^ Moreover, Wnt signalling has been correlated to congenital diseases and cancers, as well as indicating that miR‐140‐5p plays a significant role in the regulation of Wnt signalling.^20^, ^22^ Mayorga et al. 26 pointed out that miR‐145 expression could be used as a regulator of activity of β‐catenin in terms of hypoxia and ischaemia. Moreover, miR‐140‐5p could inhibit angiogenesis in a rat model of ischaemia by targeting VEGFA, which may be beneficial for cerebral ischaemia treatment.^8^ Additionally, it was demonstrated during our study that the mRNA and protein expressions of Wnt1, β‐catenin, TCF‐4 and E‐cadherin were increased in other groups as compared with the model group. β‐catenin/TCF‐4 mutations regulating Wnt signalling and E‐cadherin gene have been linked with the development of brain oncogenesis.^27^ Wnt1 has been proven to protect against neuronal injury, protein of which significantly increases neuronal cell survival.^28^ Furthermore, β‐catenin with TCF could activate some specific target genes related to cell apoptosis, and increased TCF‐4 mRNA expression is helpful for survival of breast cancer patients.^29^ Consistent with the aforementioned finding, a previous study asserted that overexpressed β‐catenin could inhibit apoptosis induced by hypoxia through the HIF‐1α signalling, suggesting that mRNA and protein expression of β‐catenin and TCF‐4 may be up‐regulated in HIBD rats.^30^

The article "MicroRNA‐140‐5p elevates cerebral protection of dexmedetomidine against hypoxic–ischaemic brain damage via the Wnt/β‐catenin signalling pathway" was retracted in 2021. Reasons: fabricated or falsified data; manipulated images; an official misconduct investigation; misconduct by an author.

In addition, our study showed that the combined action of DEX and miR‐140‐5p has protective effects on HIBD in neonatal rat brains, which could reduce neuronal apoptosis in hippocampus of rats. Although DEX or miR‐140‐5p mimic alone also exhibited protection against hypoxic–ischaemic brain damage, the DEX + miR‐140‐5p mimic group showed more significant difference in the above figures. As a potent and selective alpha‐2 agonist, DEX has a neuroprotective effect on hippocampus and dentate gyrus, similar to that in this study.^31^ DEX can be used as a therapeutic drug for treating HIBD and promoting functional recovery after ischaemia.^32^, ^33^ Rats with ischaemia/reperfusion (I/R) treated with DEX were shown to have decreases in relation to their neurological deficit scores, cerebral infarct volume, brain oedema and neuron death in the CA1 region of hippocampus and cortex area, suggesting that the apoptosis rate may be down‐regulated.^34^, ^35^ Studies have held the position that HI could lead to neuronal cell death and neuronal damage, and apoptosis is essential in HI damage of the neonatal brain.^36^, ^37^ HI damage in the hippocampus is more sensitive than that in other brain regions, and HI damage results in the death of many neurons, through the vehicle of both the processes of apoptosis and necrosis.^38^ In our study, we found that the weight and length growth, weight ratio of the left hemisphere to the right hemisphere and the rate of reaching standard were all increased; however, decreases were recorded for total response times, total response duration and neuronal apoptosis rate in the hippocampus, when HIBD rats had been treated with DEX + miR‐140‐5p mimics or si‐Wnt1. A previous study has demonstrated that miR‐140‐5p inhibits the MAPK signalling pathway in hepatocellular carcinoma.^39^ DEX has also been demonstrated to protect the brain against isoflurane‐induced neuroapoptosis in the hippocampus of neonatal rats by suppressing the p38MAPK signalling pathway.^40^ However, the side effects of DEX have also been indicated that DEX infusion results in mild analgesia, reversible sedation and memory impairment which may decrease central nervous system activity.^41^ So, DEX added with miR‐140‐5p mimic serves as a better treatment regimen than DEX infusion alone. Bcl‐2 protein, the key mediator of mitochondrial pathway, has been determined to play an essential role in apoptosis and ischaemic neuronal death, and Bcl‐2 expression could be increased by DEX, which again was largely consistent with the findings of our study.^42^, ^43^ Bax, belonging to the Bcl‐2 family, has been discovered that its inhibitory peptide reduces apoptosis in neonatal rat hypoxic–ischaemic brain damage, which is inhibited by DEX.^42^, ^44^

In conclusion, by targeting Wnt1 through the negative regulation of the Wnt/β‐catenin signalling pathway, miR‐140‐5p abated neuron apoptosis in the hippocampus and resulted in reductions in the death rate of neonatal rats with HIBD; more importantly, miR‐140‐5p was shown to enhance the cerebral protection role of DEX from HIBD in neonatal rats. Although these results provide validation, the research findings translating into clinical application still need to be verified. Moreover, the specific and inner mechanism of DEX influencing HIBD is not yet defined. Further empirical researches are needed to transfer the therapeutic values of miR‐140‐5p to clinical care in the treatment of HIBD.

## COMPETING INTERESTS

The authors have declared that no competing interests exist.
